# Early Identification of High-Risk Factors for Upper Gastrointestinal Bleeding

**DOI:** 10.1155/2022/5641394

**Published:** 2022-10-13

**Authors:** Xuesong Jin, Xiaohong Wang, Pengfei Mao

**Affiliations:** Department of Gastroenterology, Suzhou Hospital of Integrated Traditional Chinese and Western Medicine, Jiangsu 215101, China

## Abstract

**Objective:**

To identify simple and accurate pre-endoscopy risk factors for early identification of high-risk upper gastrointestinal bleeding.

**Methods:**

Patients who were admitted to Suzhou Hospital of Integrated Traditional Chinese and Western Medicine from January 1, 2016, to December 31, 2019, due to upper gastrointestinal bleeding were retrieved, and the detailed clinical data of the above patients were collected. Patients with a definite diagnosis of bleeding from esophageal/and gastric varices were assigned to the high-risk group. Patients with bleeding not caused by varices were divided into a high-risk and a low-risk group according to the Forrest grading and scoring standard (high-risk group Forrest Ia-IIb, low-risk group Forrest IIc-III). Univariate analysis, *t*-test, chi-square test, binary logistic regression, ROC curve (Receiver-operating characteristic curve), etc. were employed for analysis in order to identify some simple and accurate risk factors for high-risk upper digestion tract bleeding before endoscopy.

**Results:**

A total of 916 patients were collected. Three risk factors among the screened risk factors (1) hemoglobin ≤ 85 g/L, (2) vomiting red blood, and (3) “red bloody stool” were analyzed by ROC curve analysis. The specificities of each factor were 78.4%, 94.5%, and 96.7%, respectively, and the sensitivities were 71.8%, 55.9%, and 23.1%, respectively. We also derived a risk prediction scoring system for the three factors that meet the high risk such as (1) hemoglobin ≤ 83 g/L, (2)vomiting red blood, and (3) “red bloody stool.” The area under the ROC curve (AUROC), sensitivity, and specificity were 0.877, 0.904, and 0.746.

**Conclusion:**

Hemoglobin ≤ 85 g/L, vomiting red blood, and red bloody stool were included in a simple scoring standard for predicting high-risk UGIB patients before endoscopy. The new risk prediction scoring system requires only three indicators and has the advantages of high accuracy, short time-consuming, and easy application.

## 1. Introduction

Acute upper gastrointestinal bleeding (AUGIB) refers to the bleeding above the ligament of Trevor's, the main clinical manifestations are hematemesis, melena, etc. It is a common and potentially life-threatening emergency clinical disease. Its annual incidence rate is (100–180)/100,000 [1]. Among them, nonvariceal upper gastrointestinal bleeding accounts for the vast majority, about 80%–90%, and variceal bleeding accounts for about 10% [2]. Although variceal bleeding is a minority among all upper gastrointestinal bleeding (UGIBs), it has a high mortality rate of 30 percent in initial hospitalization, nearly 60 percent within 1 year [3], and rebleeding occurs in 70 percent of patients [4]. In patients with nonvariceal bleeding such as high-risk ulcer Forrest Ia, the rebleeding rate is as high as 90% [5]. The management and timing of endoscopy in patients with high-risk conditions in UGIB differs from other patients because it predicts higher rates of rebleeding and mortality [6]. Therefore, risk stratification is important for determining treatment indications and predicting clinical outcomes, and early identification of high-risk patients is essential for intensive treatment and early intervention. At present, many studies have shown that endoscopy is key to the diagnosis of upper gastrointestinal bleeding, and it is also the gold standard for identifying active bleeding. Drug combined with endoscopy is now the preferred treatment, no matter in variceal bleeding or nonvariceal bleeding [7, 8]. More studies have shown that advanced endoscopic therapy can significantly reduce the rebleeding rate and mortality of patients with gastrointestinal bleeding, and improve the prognosis of patients [9]. Currently widely accepted pre-endoscopy scoring systems are Glasgow Blatchford Score (GBS), Rockall Score (RS), and AIMS65. Among them, GBS has a high predictive value in terms of intervention and mortality [10]. However, these criteria are complicated to calculate or need to be completed after endoscopy before further evaluation, making it difficult to apply them clinically. A study found that only about 50% of the surveyed 1,000 related doctors knew about these scoring systems, and 30% of them had used one of these scoring systems for patients with UGIB [11]. To date, there is no universally agreed scoring standard for predicting high-risk upper gastrointestinal bleeding populations, and the existing scoring systems have not been updated to adapt to changes in clinical characteristics. Our purpose is to screen out high-risk UGIB patients using a more accurate, simple, and convenient scoring standard, which reminds clinicians to take the next step of diagnosis and treatment as soon as possible.

## 2. Materials and Methods

Admitted patients were retrieved from the Gastroenterology Department of Suzhou Integrated Traditional Chinese and Western Medicine Hospital from September 1, 2016, to September 30, 2018. The included patients should have symptoms of active hematemesis or melena, with the gastroscopy-confirmed presence of explainable lesions leading to upper gastrointestinal bleeding. Endoscopy should be completed within 24–48 hours after admission. Exclude patients who were unwilling to take endoscopy or had malignant diseases, hematological disorders, mental illness, drug allergies, etc.

Detailed medical history, such as cardiovascular and cerebrovascular diseases, liver cirrhosis, hypertension, diabetes, recent drug (NSAIDs, hormone drugs) taking history, etc. were collected. Clinical manifestations included the color of hematemesis, the color of stool, cold sweat, palpitations, and syncope. Vital signs included systolic blood pressure, diastolic blood pressure, and heart rate.

The laboratory data of UGIB patients within 48 hours of hematemesis or melena were collected for analysis, including prothrombin time (PT), activated partial prothrombin time (APTT), hemoglobin (Hb), hematocrit (MCV), the lowest value of platelet count (PLT), the highest value of blood urea nitrogen (BUN), and serum creatinine (SCr).

Endoscopy results: gastroscopy should be performed within 24–48 hours after symptoms appear, and those with peripheral circulatory failure should be corrected first. Endoscopy includes evidence of esophageal and gastric variceal bleeding such as (1) active bleeding from varices; (2) “white papilla” overlying varices; and (3) variceal overlying blood clots or no other Varicose veins that are the underlying cause of bleeding. For nonvariceal bleeding, the Forrest grading scale was used. All endoscopic diagnostic criteria were jointly decided by three endoscopists. Patients were treated according to the consensus of the Asia-Pacific Working Group recommended by the international consensus [12]. The standard of care is as follows: start PPIs like pantoprazole, omeprazole, and esomeprazole for all patients with upper GI bleeding who are admitted to the hospital. Blood transfusion is required in the following situations: the patient presents with unstable hemodynamics, such as systolic blood pressure <90 mmHg, heart rate > 120 beats/min, and hemoglobin < 70 g/L. Principles of endoscopic treatment: the treatment of acute esophageal variceal bleeding (EVB) mainly includes conservative drug administration, endoscopic treatment, balloon tamponade, transjugular intrahepatic portal shunt (TIPS), and surgical treatment [13]. For nonvariceal upper gastrointestinal bleeding, submucosal injection of epinephrine, electrocoagulation, titanium clips, or a combination of these methods are used alone. Patients with esophageal and gastric varices are treated with endoscopic band ligation, tissue adhesive injection, combined treatment with multiple methods, and interventional surgery, which depends on the judgment of the endoscopic surgeon [14].

### 2.1. Statistical Methods

SPSS17.0 (Armonk, NY) was used for statistical analysis and processing of data. The description of measurement data was performed by mean + standard deviation (*X* ± SD), and the description of categorical variable data was performed by percentage. Univariate factor analysis was performed for measurement data using an independent samples *t*-test, and the chi-square test was used for categorical variable data. The factors with significant significance between the two groups of data were included in the binary logistic regression analysis, and the relevant high-risk factors were obtained. Then the obtained high-risk factors were combined to establish a regression equation model (inclusion level 0.05, exclusion level 0.10). The independent risk factors screened above were compared individually and also in combination. Statistically significant was set at a two-sided *P* < 0.05.

## 3. Results

### 3.1. Clinical Characteristics of 916 UGIB Patients

A total of 1079 UGIB patients were retrieved, of which 108 patients underwent endoscopic examination more than 48 hours beyond the initial bleeding, 53 patients had chronic anemia, and 2 patients had bleeding in other parts of the upper gastrointestinal tract (1 patient with biliary bleeding, 1 patient with pancreatic cancer involving duodenum hemorrhage). The remaining 916 patients with upper gastrointestinal bleeding were included in this study, and 372 patients were at high risk according to the Forrest classification, accounting for 40.61% of the study population. Among them, there were 17 Forrest Ia patients (4.57%); 56 Forrest Ib patients (15.05%), 205 Forrest IIa patients (55.11%), and 94 Forrest IIb patients (25.27%). There were 425 low-risk patients, accounting for 46.39% of the study population, including 74 Forrest IIc patients (8.08%) and 351 Forrest III patients (34.39%). There were 119 patients with EVB bleeding, accounting for 12.99% of the study population. Due to the high recurrence rate and mortality rate of bleeding caused by EVB [15, 16], they were all included in the high-risk group. In summary, there were 491 patients in the high-risk group and 425 in the low-risk group. The average age of the patients was 57.13 ± 17.31 years old in the high-risk group, and 52.54 ± 18.19 years old in the low-risk group (*P* < 0.05). The ratio of males to females was 195 : 296 in the high-risk group, and 112 : 313 in the low-risk group (*P* < 0.05), as shown in Table 1. The etiology of UGIB in this study included peptic ulcer in 813 cases (88.76%), a gastrointestinal tumor in 33 cases (3.60%), dieulafoy ulcer in 14 cases (1.53%), acute erosive hemorrhagic gastritis in 11 cases (1.20%), and cardiac tear in 45 cases (4.91%).

Among the 916 patients, there were significant differences between the two groups in terms of previous underlying diseases, non-steroidal anti-inflammatory drugs use, hepatitis, liver cirrhosis, and hypertension (*P* < 0.05). Clinical manifestations include “vomiting red blood, red bloody stools, and shock,” “diastolic blood pressure” in vital signs, and “prothrombin time, activated partial thromboplastin time, hemoglobin, hematocrit” in laboratory hematology indexes, platelet count, albumin,” which had statistical differences between the two groups (*P* < 0.05). It is suggested that the above 16 indicators may be meaningful for predicting high-risk UGIB patients. The 16 factors were further analyzed below, and the specific data are shown in Table 1.

### 3.2. Logistic Analysis of Clinical and Laboratory Characteristics for High-Risk UGIB Patients

Further binary logistic regression analysis was performed on the 8 meaningful categorical variables of “gender, non-steroidal anti-inflammatory drugs use, hepatitis, liver cirrhosis, hypertension, vomiting red blood, solution of red bloody stool, and shock.” The five indicators of “gender, liver cirrhosis, vomiting red blood, red bloody stool, and shock” (*P* < 0.05) were risk factors for high-risk UGIB patients, and their odds ratios were 0.582, −1.877, 3.058, 2.215, and 0.855. Logit = −19.326 + 0.582 × gender − 1.877 × cirrhosis + 3.058 × vomiting red blood + 2.215 × red bloody stool + 0.855 × shock. The Cox and Snell *R*^2^ was 0.434, and the Nagelkerke *R*^2^ was 0.580.

Further binary logistic analysis was performed on the 8 indicators of meaningful measurement variables of “age, diastolic blood pressure, prothrombin time, activated partial prothrombin time, hemoglobin, hematocrit, platelet count, albumin,” and only hemoglobin, hematocrit, platelet, prothrombin time, and albumin were statistically significant (*P* < 0.05), which were regarded as risk factors for high-risk UGIB patients, with odds ratios of 0.891, 1.259, 0.995, 1.112, and 0.963. Logit = 4.501 – 0.115 × hemoglobin + 0.230 × hematocrit − 0.005 × platelet + 0.106 × prothrombin time − 0.037 × albumin. The Cox and Snell *R*^2^ was 0.328, and the Nagelkerke *R*^2^ was 0.438 (Table 2).

### 3.3. Logistic and ROC Analysis of Clinical and Laboratory Characteristics for High-Risk UGIB Patients

The 10 indicators of “gender, liver cirrhosis, vomiting of red blood, solution of red bloody stool, shock, hemoglobin, hematocrit, platelet, prothrombin time, and albumin” were combined and further analyzed, and the results showed that gender, shock, red blood cell pressure, the partial regression coefficients of blood clots, platelets, prothrombin time, and albumin were statistically significant (*P* < 0.05). Finally, three indicators of “liver cirrhosis, vomiting of red blood, solution of red bloody stool, and hemoglobin” were used as high-risk factors for predicting high-risk UGIB. The regression equation was: Logit = 2.136 + −0.018 × hemoglobin + 2.812 × vomiting red blood + 1.673 × relieving red bloody stool, Cox & Snell *R*^2^ was 0.405, Nagelkerke *R*^2^ was 0.550, and the detailed data are shown in Table 3.

The “hemoglobin” was used to make the ROC curve according to the risk level of VUGIB. The optimal critical value of hemoglobin was 85 g/L, and the specificity, sensitivity, positive likelihood ratio, negative likelihood ratio, Youden index, and AUROC were 0.772, 0.774, 3.395, 0.293, 0.546, 0.820 (*P* < 0.05) are shown in Figure 1 and Table 4.

The ROC curve evaluation of the four indicators of hemoglobin ≤ 85 g/L, vomiting of red blood, solution of red bloody stool, and history of liver cirrhosis showed that the sensitivity of the three were 0.772, 0.651, 0.255, and 0.329, and the specificity was 0.772, 0.651, 0.255, and 0.329.0.771, 0.936, 0.962, 0.979, AUROC were 0.772, 0.794, 0.608, 0.654.

The four high-risk factors screened above were further defined as “(1) hemoglobin ≤ 85 g/L, (2) red blood vomiting, (3) red bloody stool, and (4) history of liver cirrhosis”, and the vomit color was “bright red, dark red or with “blood clot” is defined as 1 point, other is 0 point; stool color is “bright red, dark red or accompanied by blood clot” is defined as 1 point, other is defined as 0 points; hemoglobin ≤ 83 g/L is defined as 1 point scores, otherwise defined as 0 points; and history of liver cirrhosis defined as 1 point, otherwise defined as 0 points. Combinations of ①②, ①③, ①②③, and ①②③④ were constructed to form four risk prediction scoring systems, e.g., score1, score2, score3, and score 4, respectively. The Blatchford scoring system and the resulting new scoring systems were evaluated by the ROC curve. When the critical value was 0.5, the maximum ROC curve area was 0.877, the sensitivity was 0.904, the specificity was 0.746, and the Youden index was 0.650 (*P* < 0.05). The *P* values, sensitivity, specificity, and cutoff points of the two scoring systems and the BRS scoring system are shown in Figure 1(c)and Table 4.

A correlation analysis by Wuerth and Rockey [17] found that after 72 hours of successful endoscopic hemostasis, Forrest Ib had a very low rebleeding and rebleeding rate compared with Forrest Ia, Forrest IIa, and Forrest IIb patients. Therefore, we eliminated the 33 participants who were classified as Forrest Ib and passed them through univariate analysis (*t*-test, chi-square test), binary logistic regression, and ROC curve again, and still obtained “(1) vomiting red blood, (2) Red bloody stool, and (3) hemoglobin≤85 g/L” were three high-risk factors, and a new scoring system ①③ and ①②③ were constructed to form two risk prediction scoring systems of score3 and score4, respectively. The Blatchford scoring system and the resulting new scoring system were evaluated by the ROC curve. See Figure 1 and Table 3 for details.

## 4. Discussion

AUGIB refers to bleeding caused by diseases of the gastrointestinal tract above the ligament of Trevor, including pancreatic or bile duct bleeding and bleeding caused by diseases near the anastomotic stoma after gastrojejunostomy [15]. Due to advanced medical and endoscopic treatment, the hospitalization rate for upper gastrointestinal bleeding has decreased by 20% in the past decade, and the mortality rate has dropped from 4.5% to about 2.1%. Although the hospitalization rate and case fatality rate have decreased, the number of people is still larger for a larger population base. In fact, patients with variceal bleeding are considered a specific high-risk group [18]. Due to the high mortality rate and many complications of esophageal and gastric variceal bleeding, early identification of high-risk patients is extremely important, so it still has great research value.

In fact, patients with variceal bleeding are considered a specific high-risk group. A study by Cho SH [19] compared patients undergoing emergency endoscopy with regular gastroscopy, and there were significant differences in mortality, blood transfusion volume, and need for clinical intervention. Therefore, early identification of high-risk UGIB patients and early improvement of endoscopy can further improve the prognosis of patients. At present, a variety of scoring systems have been clinically used to assess the risk of upper gastrointestinal bleeding, each of which has different specificity, sensitivity, and predictive value for clinical observation indicators. The most commonly used risk assessment systems are the Forrest classification [20], BRS scoring standard, AIMS56 [21], and Rockall score, each of which has the characteristics of complex calculation and/or the need for endoscopy results, which makes the risk assessment system more complex for clinical application [20]. At present, researchers have proposed that accurate prediction of a series of risks in patients with UGIB is helpful for clinically selective management of these patients, and it is recommended that risk assessment should classify patients into high-risk and low-risk, because this may help clinicians make early decisions, such as the choice of endoscopy time, patient allocation, choice of level of care, and time to leave the hospital [22]. Early identification and evaluation of high-risk patients can improve the effectiveness of clinical treatment, shorten the time of treatment for patients, reduce the cost of treatment for patients, and improve clinical outcomes for patients.

Endoscopy is the key to diagnosing the etiology of upper gastrointestinal bleeding, and drug combined with endoscopy is now the preferred treatment [23]. Studies have shown that there is no solid basis for the benefit of earlier endoscopy. The Forrest classification has been used to identify high-risk endoscopic nonvariceal upper gastrointestinal bleeding. The Forrest grading is based on the results of endoscopy. Since the Forrest grading can better predict the risk of UGIB rebleeding, it can more intuitively determine which UGIBs really need endoscopic intervention [24]. We took the Forrest classification as the gold standard for judging the severity of UGIB and divided UGIB patients into high-risk groups and low-risk groups according to the actual Forrest classification. The etiological analysis was consistent with the common etiology reported by the guideline [25]. We determined “hemoglobin” by ROC curve analysis, and the optimal critical value of hemoglobin was 83 g/L (see Table 4 and Figure 1(a) for details). Several clinical studies have suggested that hemoglobin between 80 and 85 g/L is a high-risk factor for acute upper gastrointestinal bleeding [5], and the conclusions drawn by our study were consistent with this. In the study of Forrest et al. [26], “vomiting bright red blood” was one of the high-risk indicators.

According to the correlation analysis by Zaragoza et al. [20], even after we excluded 33 participants who were classified as Forrest Ib, and through the aforementioned similar statistical methods, we still concluded that “(1) vomiting red blood, (2) red bloody stool, and (3) hemoglobin≤ 83 g/L” were three high-risk factors, and a new scoring system ①③ and ①②③ were constructed to form two risk prediction scoring systems of score3 and score4, respectively. It can be seen from Figure 1(d) that among the two newly constructed risk prediction scoring systems, the risk prediction score 3 has the largest AUROC area of 0.871 when the critical value is 0.5, and the sensitivity, specificity, and Youden index were 89.8%, 75.4%, and 75.4%, respectively. When the critical value of scoring system 4 was 0.5, the AUROC area was 0.885, and the sensitivity, specificity, and Youden index were 92.0%, 74.6%, and 0.665, respectively. The Blatchford scoring system and the new scoring system were used to evaluate the ROC curve, and the results showed that the above two scoring systems were better than BRS, score1, and score2 in evaluating patients with the high-risk nonvariceal upper gastrointestinal bleeding system. The value of our scoring system should be evaluated in severe cases, such as fulminant hepatitis, inflammation, infections, hypoxia, or preterm birth [27–37].

In conclusion, this study showed that “hemoglobin ≤ 83 g/L, vomiting red blood, and red bloody stool” could be three independent high-risk factors in patients with UGIB, while the combined application of these three risk factors can be a good way to screen high-risk UGIB patients before endoscopy.

## Figures and Tables

**Figure 1:** ROC curve of risk factors.

**Table 1:** Clinical characteristics of 916 UGIB patients.

Clinical factors	Low risk (*n* = 425)	High risk (*n* = 491)	*P*
Gender, male	112 (26.35%)	195 (39.71%)	< 0.001
Age, *y*	52.54 ± 18.19	57.13 ± 17.31	< 0.001
SBP (mmHg)	121.61 ± 17.37	119.32 ± 20.85	0.083
DBP (mmHg)	73.55 ± 11.32	69.00 ± 12.54	< 0.001
HR (beat/min)	85.12 ± 14.06	83.93 ± 16.92	0.077
Hb (g/L)	100.49 ± 21.88	73.63 ± 20.71	< 0.001
HCT (%)	30.09 ± 6.73	22.73 ± 6.12	< 0.001
PLT (*∗* 10^9)	198.26 ± 61.33	151.40 ± 81.45	< 0.001
PT (s)	13.62 ± 2.35	15.22 ± 2.94	< 0.001
APTT (s)	32.38 ± 9.21	34.69 ± 7.81	< 0.001
Albumin (g/L)	36.68 ± 5.34	31.06 ± 9.52	< 0.001
BUN (mmol/L)	10.29 ± 6.79	11.95 ± 3.14	0.115
Cr (umol/L)	73.23 ± 24.01	78.76 ± 75.04	0.146
NSAID	21.88%	15.89%	0.022
Corticosteroids	0.47%	1.63%	0.116
Liver cirrhosis	5.41%	18.33%	< 0.001
Hypertension	31.16%	41.88%	0.001
Hepatitis	2.11%	33.40%	< 0.001
Diabetes mellitus	13.65%	17.31%	0.144
Cardiovascular diseases	12.47%	10.79%	0.496
Weight loss	4.24%	2.65%	0.203
Red hematemesis	6.36%	64.77%	< 0.001
Red stool	3.76%	25.25%	< 0.001
Palpation	48.71%	50.92%	0.508
Cold sweat	42.12%	48.27%	0.063
Syncope	16.00%	16.29%	0.928
Shock	2.82%	12.83%	< 0.001

APTT = activated partial thromboplastin time; BUN = blood urea nitrogen; DBP = diastolic blood pressure; Hb = hemoglobin; HCT = hematocrit; HR = heart rate; NSAIDs = non-steroidal anti-inflammatory drugs; PLT = platelet cell; PT = prothrombin time; SBP = systolic blood pressure.

**Table 2:** Logistic analysis of clinical and laboratory characteristics for high-risk UGIB patients.

Characteristics	Equation	Cox and Snell *R*^2^	Nagelkerke *R*^2^	Exp (*R*^2^)	*P*
Sex	−19.326 + 0.582 × sex − 1.877 × cirrhosis + 3.058 × red hematemesis × +2.215 × red stool + 0.855 × shock	0.434	0.580	0.582 (sex) −1.877(cirrhosis) 3.058 (hematemesis) 2.215 (red stool) 0.855 (shock) −1.433 (constant)	< 0.001 (hematemesis) < 0.001 (red stool) 0.012 (shock) < 0.001 (constant)
NSAID					
Corticosterioids					
Hepatitis					
Cirrhosis					
HBP					
Diabetes mellitus					
Cardiovascular disease					
Red hematemesis					
Red stool					
Weight loss					
Palpation					
Cold sweat					
Syncope					
Shock					
Age	4.501 – 0.115 × Hb + 0.230 × HCT + 0.005 × PLT + 0.106 × PT-0.0.037 × Albumin	0.328	0.438	0.891(Hb) 1.259 (HCT) 0.995 (PLT) 1.112 (PT) 0.963 (albumin) 3.055 (constant)	<0.001 (Hb) <0.001 (HCT) <0.001 (PLT) 0.048 (PT) 0.028 (albumin) < 0.001 (constant)
SBP					
DBP					
HR					
Hb					
HCT					
PLT					
PT					
APTT					
Albumin					
BUN					

APTT = activated partial thromboplastin time; BUN = blood urea nitrogen; DBP = diastolic blood pressure; Hb = hemoglobin; HCT = hematocrit; HR = heart rate; NSAID = non-steroidal anti-inflammatory drug; PLT = platelet cell; PT = prothrombin time; SBP = systolic blood pressure.

**Table 3:** Logistic analysis of clinical and laboratory characteristics for high-risk UGIB patients.

Risk	ß	Exp (*ß*)	*P*	Cox & Snell *R*^2^	Nagelkerke *R*^2^
Red hematemesis	3.113	22.483	< 0.001	0.4498	0.665
Red stool	1.795	6.020	< 0.001		
Hb	−0.083	0.920	< 0.001		
Cirrhosis	1.449	4.259	0.002		

^*∗*^ Hb = hemoglobin.

**Table 4:** ROC analysis of clinic and laboratory for characteristics for high-risk UGIB patients.

Scoring system	Cutoff point	*P*	AC	Sensitivity	Specificity	PLR	NLR	Youden index
Hb (g/L)	85	< 0.001	0.820	0.744	0.772	3.395	0.293	0.546
Hb ≤ 85 (g/L)	0.5	< 0.001	0.772	0.772	0.771	3.371	0.296	0.543
Red hematemesis	0.5	< 0.001	0.794	0.651	0.936	10.172	0.373	0.587
Red stool	0.5	< 0.001	0.608	0.255	0.962	6.711	0.774	0.217
Liver cirrhosis	0.5	< 0.001	0.654	0.329	0.979	15.667	0.685	0.307
SCORE1	0.5	< 0.001	0.885	0.932	0.738	0.557	0.092	0.670
	1.5	< 0.001		0.491	0.969	15.839	0.525	0.460
SCORE2	0.5	< 0.001	0.830	0.817	0.757	3.362	0.242	0.574
	1.5	< 0.001		0.209	0.976	8.780	0.810	0.186
SCORE3	0.5	< 0.001	0.900	0.959	0.726	3,500	0.056	0.685
	1.5	< 0.001		0.589	0.948	11.327	0.433	0.537
	2.5	< 0.001		0.129	0.995	25.800	0,875	0.125
SCORE4	0.5	< 0.001	0.911	0.961	0.715	3.372	0.055	0.676
	1.5	< 0.001		0.659	0.941	11.169	0.362	0.600
	2.5	< 0.001		0.326	0.993	46.571	0.679	0.319
	3.5	< 0.001		0.060	1.000	—	0.940	0.060
Blatchford score		< 0.001						
		< 0.001						
		< 0.001						

Hb = hemoglobin; UGIB = upper gastrointestinal bleeding; PLR = positive likelihood ratio; ROC = receiver-operating characteristic.

## Data Availability

The data used to support the findings of this study are available from the corresponding author upon request.
